This article has been retracted.

# Clinical Value of Three-Dimensional Transvaginal Ultrasound in Diagnosis of Endometrial Receptivity and Ovarian Function in Patients with Infertility

**DOI:** 10.1155/2022/8438131

**Published:** 2022-05-11

**Authors:** Jingjing Wu, Xiangming Zhu, Junjun He, Caihong Ye, Bo Pang, Tianying Zhao, Tingting Bao

**Affiliations:** ^1^Ultrasonics, Yi Jishan Hospital, Wannan Medical College, Wuhu 241000, China; ^2^Anesthesiology Department, Wuhu Fifth People's Hospital, Wuhu 241000, China

## Abstract

**Objective:**

A case-control study was conducted to explore the clinical value of three-dimensional transvaginal ultrasound in the diagnosis of endometrial receptivity (ER) and ovarian function in patients with infertility.

**Methods:**

A total of 308 infertile women treated in our hospital from March 2020 to June 2021 were enrolled as the observation group, and another 300 women of childbearing age who underwent physical examination in the same period were enrolled as the control group. The clinical value of three-dimensional transvaginal ultrasound in ER in patients with infertility was analyzed by comparing the classification of endometrial and subendometrial blood perfusion, endometrial AUC value and Pi value, and subendometrial AUC value and Pi value. According to the number of oocytes obtained, the patients were assigned into the normal response group (182 cases, ≥5 oocytes) and the low response group (126 cases, <5 oocytes). The levels of some hormones, such as follicle-stimulating hormone (FSH), luteinizing hormone (LH), estradiol (E2), and FSH/LH, were measured. Transvaginal ultrasonography was performed to detect ovarian volume (OV), antral follicle count (AFC), and peak flow rate of the ovarian interstitial artery (PSV). The peak of end-diastolic flow velocity (EDV) and other indexes were analyzed. The correlation between FSH level, FSH/LH, and ultrasound indexes was analyzed, and the ROC curve was established to analyze the value of transvaginal Doppler ultrasound in evaluating ovarian reserve function and predicting ovulation.

**Results:**

There were significant differences in late proliferation type I and type III, ovulatory type II and type III (*P* < 0.05). There exhibited no significant difference in late proliferation type II, ovulation stage type I, and implantation window stage type I, type II, and type III (*P* > 0.05). Regarding the endometrial AUC and Pi values, the endometrial AUC and Pi values in the observation group were lower compared to the control group during late proliferation and ovulation (*P* < 0.05). There exhibited no significant difference in AUC and Pi (*P* > 0.05). Regarding the subintimal AUC and Pi values, the subintimal AUC and Pi values in the observation group were higher compared to the control group during late proliferation and ovulation (*P* < 0.05). There exhibited no significant difference in AUC and Pi during the implantation window (*P* > 0.05). There exhibited no significant difference in menarche age, age, body mass index, and menstrual cycle between the normal response group and the low response group (*P* > 0.05). The levels of EDV, OV, AFC, and PSV in the normal response group were higher compared to the low response group (*P* < 0.01). Compared with the low response group, the levels of FSH and FSH/LH in the normal response group were lower, but the levels of LH and E2 in the normal response group were higher (*P* < 0.05). The results of correlation analysis of FSH, FSH/LH, and ultrasound parameters between the normal response group and the low response group indicated that FSH was negatively correlated with E2, EDV, OV, AFC, and PSV in 308 infertile women (*r* = −0.817, -0.846, -0.707, -0.845, -0.911, *P* < 0.01), but it was positively correlated with FSH/LH (*r* = 0.714, *P* < 0.01). The ultrasound parameters of ovarian reserve function in the normal response group and the low response group were compared with the indexes that predicted ovulation. The results of ROC curve analysis indicated that the cutoff values of EDV, OV, AFC, and PSV were 4.141, 3.726, 4.106, and 13.944, respectively, the specificity of each index was higher than 90.00%, and the sensitivity was higher than 80.00% except PSV.

**Conclusion:**

Transvaginal ultrasound can not only accurately evaluate the ER of infertile women but also directly observe follicular development and monitor ovulation, which is of high value in evaluating ovarian reserve function and predicting ovulation.

## 1. Introduction

Infertility refers to a kind of disease in which the normal sexual life is cohabited for more than 1 year without any contraceptive measures, and the female does not become pregnant or cannot maintain pregnancy [1]. Infertility is a global thorny medical problem, which not only seriously affects the quality of life of husband and wife, family happiness, but also involves the national medical level, reproductive health, and other issues [2]. The incidence of infertility in China is 7% to 10%, among which the incidence of women is increasing year by year. Abnormal endometrium, tubal adhesion, and ovulation dysfunction can lead to female infertility, of which the proportion of infertility caused by abnormal ovulation function is the highest, so monitoring ovulation is particularly important for the clinical diagnosis and treatment of infertility [3].

Infertility is divided into primary infertility and secondary infertility, the former refers to never getting pregnant, and the latter refers to having been pregnant but infertile, which is usually the main factor affecting most female infertility is ovulation dysfunction [4]. At present, the evaluation of ovarian reserve function mainly depends on basic endocrine hormone determination and ultrasound examination. Ultrasound has the advantages of nonradiation, nontrauma, and high repeatability. The routine examination can only detect whether the woman is pregnant but cannot accurately detect whether the reproductive system is pathological changes, and three-dimensional ultrasound can directly reflect the location of the lesions, so as to judge and diagnose [4, 5]. The three-dimensional ultrasound automatic volume measurement (SonoAVC) software of transvaginal three-dimensional ultrasound can automatically obtain the number, size, and volume of antral follicles. Every follicle is marked with the different colors and will not be measured repeatedly. Compared with two-dimensional ultrasound, it takes less time and is more effective [5].

Three-dimensional power Doppler ultrasound combined with virtual organ computer-aided analysis (VOCAL) software is more accurate in measuring OV [6]. VOCAL technology used a three-dimensional reconstruction method to detect and automatically calculate the ovarian vascular index, blood flow index, vascularized blood flow index, three-dimensional and intuitive display of the ovarian vascular tree, and objective and quantitative evaluation of ovarian blood perfusion [7]. In terms of color Doppler, it has no angle dependence, is easy to detect tiny blood vessels and low-speed blood flow, and can comprehensively analyze the blood supply of the whole ovary [8]. In recent years, transvaginal three-dimensional ultrasound has been deeply studied in the diagnosis of ovulatory-dysfunction infertility [9, 10]. It is found that transvaginal three-dimensional ultrasound is not affected by the shape of the reconstructed structure, exploration depth, and section. There is little difference between different examiners, so it is more accurate to evaluate the morphology, structure of ovaries, and follicles than two-dimensional ultrasound [11].

Assisted reproductive technology (ART) has become an important means for the treatment of infertility. Although the techniques of ovulation induction, embryo culture in vitro, and preimplantation genetic screening (PGS) have been continuously promoted, the embryo implantation rate of ART has not been significantly improved, and there are many factors that affect the outcome of pregnancy [12]. It mainly includes factors such as embryo quality, endometrial receptivity (ER), and synchronization between embryo and endometrium, among which ER is an important influencing factor. ER means that the endometrium in a special state allows blastocyst adhesion, penetration, and implantation, which leads to embryo implantation [13]. It is generally believed that endometrial pathological biopsy is the gold standard for its evaluation, but its clinical application is limited because of its invasiveness [14, 15]. Ultrasound is more widely employed in the evaluation of ER. Based on this, this paper discusses 308 infertile women treated in our hospital from March 2016 to June 2021, which are reported as follows.

## 2. Patients and Methods

### 2.1. General Information

A total of 308 infertile women treated in our hospital from March 2020 to June 2021 were enrolled as the observation group, and another 300 women of childbearing age who underwent physical examination in the same period were enrolled as the control group. In the observation group, the age was 20-42 years old, and the average age was 29.18 ± 3.76 years old, and in the control group, the age was 22-44 years old, and the average age was 30.18 ± 3.54 years old. There exhibited no statistical significance in the general data. This study was permitted by the Medical Ethics Association of our hospital, and all patients signed informed consent.

The inclusion criteria are as follows: (1) women with infertility have normal sexual life for not less than 1 year; (2) women with healthy childbearing age have no gynecological diseases, normal menstruation, and have a reproductive history within 1 year; and (3) all subjects have normal understanding, expression, and communication skills and voluntarily participate in this study.

The exclusion criteria are as follows: (1) patients who took drugs that may affect pelvic blood supply 2 months before entering the group, (2) patients with a history of hematological diseases, (3) patients with gynecological diseases such as ovarian cysts, (4) patients with bilateral tubal obstruction or ovulation disorders, and (5) complicated with endometritis or pelvic infection.

### 2.2. Investigation Methods

#### 2.2.1. Evaluation of ER

Patients were examined with pulse frequency: 4~6 cm/s and probe frequency: 4~9.5 MHz. Ultrasonography was performed on the 10th to 12th day of menstruation (late proliferation), from the day of ovulation to the second day after ovulation (ovulation), and from the 8th to 10th day after ovulation (implantation window). The time of ovulation was determined according to the concentration of LH in urine and the results of transvaginal ultrasound. The median long axis section of the gray scale of the uterus was obtained, and the blood perfusion of the endometrium and subendometrium was detected by transvaginal color Doppler flow imaging (CDFI). The 5 mm of the outer margin of the endometrium was set as the subendometrial region, and the subendometrial blood flow was classified according to the blood perfusion of the endometrium and subendometrium: type I: the blood flow signal was detected in the endometrial region and close to the center of the uterine cavity; type II: the blood flow signal was detected in the endometrial region and no more than 1 cm 2 monolayer endometrium; type III: blood flow signal was detected in the subintimal area. SonoVue ultrasound contrast agent was injected into the patient's body from the patient's vein, and the median long axis section of the uterus was obtained and examined by automatic contrast-enhanced ultrasound, and the dynamic images were properly preserved. The area under the curve (AUC) and peak intensity (Pi) were analyzed by special software.

#### 2.2.2. Basic Hormone Determination

On the morning of the third day of menstrual cycle, fasting venous blood of 10 ml was isolated by centrifuge. Basic FSH, LH, and E2 were determined by automatic chemiluminescence, and the value of FSH/LH was calculated.

#### 2.2.3. Evaluation of Ovarian Function

Transvaginal Doppler ultrasound (Philips) examination: before examination, patients need to empty their bladder, take lithotomy position, use Voluson S6 color Doppler ultrasound diagnostic instrument made in the United States, and send the condom probe to the vaginal fornix or cervix to detect bilateral fallopian tubes. The monitoring began on the 3rd day of the menstrual cycle and was checked regularly every day until the follicle matured or ovulated. Ovulation standard [5]: follicles disappear or significantly decrease, follicular wall thickens and collapses, showing irregular shape, there are high-density light spots in the follicles, and the edges are serrated. Continuous monitoring can find corpus luteum images with dense light spots and thick edges. There is fluid in the Dow cavity. The number of bilateral antral follicles (AFC) was counted, the OV was calculated, and the peak flow velocity (PSV) and end-diastolic peak velocity (EDV) of the ovarian interstitial artery were measured.

### 2.3. Observation Index

The ultrasonic indexes such as EDV, OV, AFC, and PSV were compared, and the basic hormone indexes such as FSH, FSH/LH, LH, and E2 were compared.

### 2.4. Statistical Analysis

Statistical analysis was carried out by SPSS18.0 software. The counting data of endometrial and subendometrial blood perfusion classification were expressed as (%), the *χ*^2^ test was performed, and the measurement data were expressed as mean ± standard deviation (*x* ± *s*). The results of transvaginal Doppler ultrasound, basic hormone levels, AUC, and Pi were compared with an independent sample *t*-test, and the relationship between variables was analyzed by the Pearson method. The receiver operating characteristic (ROC) curve was used to analyze the transvaginal Doppler ultrasound to evaluate the ovarian reserve function and predict the value of ovulation. *P* value less than 0.05 is considered statistically significant while *P* value less than 0.01 is viewed as highly statistically significant.

## 3. Results

### 3.1. Comparison of Blood Perfusion Types of the Endometrium and Subendometrium between the Two Groups

First of all, we compared the classification of endometrial and subendometrial blood perfusion. In the observation group, there were 84 cases of late proliferative type I, 131 cases of type II, 93 cases of type III, 131 cases of type I, 83 cases of type II, and 94 cases of type III during ovulation. There were 141 cases of type I, 110 cases of type II, and 57 cases of type III in the implantation window stage. In the control group, there were 136 cases of type I, 129 cases of type II, 35 cases of type III, 136 cases of type I, 137 cases of type II, 27 cases of type III during ovulation, 125 cases of type I, 136 cases of type II, and 39 cases of type III in the control group. There were significant differences in late proliferation type I and type III, ovulation stage type II and type III (*P* < 0.05). There exhibited no significant difference in late proliferation type II, ovulation stage type I, and implantation window type I, type II, and type III (*P* > 0.05). All the results are indicated in Figure 1.

### 3.2. Comparison of the Intimal AUC Value and Pi Value between the Two Groups

We compared the intimal AUC and Pi values. The endometrial AUC and Pi values in the observation group were significantly lower compared to the control group during late proliferation and ovulation (*P* < 0.05). There exhibited no significant difference in AUC and Pi values during the implantation window (*P* > 0.05). All the results are indicated in Table 1.

### 3.3. Comparison of the Subintimal AUC and Pi Values between the Two Groups

We compared the subintimal AUC and Pi values. The subintimal AUC and Pi values in the observation group were significantly higher compared to the control group during late proliferation and ovulation (*P* < 0.05). There exhibited no significant difference in AUC and Pi values (*P* > 0.05). All the results are indicated in Table 2.

### 3.4. Comparison of General Clinical Data between the Normal Response Group and the Low Response Group

We compared the general clinical data, and there exhibited no significant difference in menarche age, age, body mass index, and menstrual cycle (*P* > 0.05). All the results are indicated in Table 3.

### 3.5. Comparison of the Results of Vaginal Three-Dimensional Ultrasound between the Normal Response Group and the Low Response Group

We compared the results of vaginal three-dimensional ultrasound examination, and the levels of EDV, OV, AFC, and PSV in the normal response group were higher compared to those in the low response group (*P* < 0.01). All the results are indicated in Table 4.

### 3.6. Comparison of Basic Hormone Levels between the Normal Response Group and the Low Response Group

We compared the basic hormone levels and the levels of FSH and FSH/LH, and the results indicated that of the normal response group were lower compared to that of the low response group, but the levels of LH and E2 in the normal response group were higher compared to those in the low response group (*P* < 0.05). All the results are indicated in Figure 2.

### 3.7. Correlation Analysis of FSH, FSH/LH, and Ultrasonic Parameters between the Normal Response Group and the Low Response Group

We analyzed the correlation between FSH and FSH/LH and ultrasonic parameters in the normal response group and the low response group. FSH was negatively correlated with E2, EDV, OV, AFC, and PSV in 308 infertile patients (*r* = −0.817, -0.846, -0.707, -0.845, and -0.911, *P* < 0.01) but positively correlated with FSH/LH (*r* = 0.714, *P* < 0.01).

### 3.8. Comparison of Ultrasonic Parameters of Ovarian Reserve Function and Indexes for Predicting Ovulation

We compared the ultrasound parameters of ovarian reserve function with the indexes of ovulation prediction. ROC curve analysis indicated that the cutoff values of EDV, OV, AFC, and PSV were 4.141, 3.726, 4.106, and 13.944, respectively, the specificity of each index was more than 90.006%, and the sensitivity was higher than 80.00% except PSV. The data are indicated in Figure 3 and Table 5.

## 4. Discussion

The results of the global big data survey show that the current incidence of infertility is relatively high, with an average of 5%-8% in developed countries, while the incidence in some backward areas of developing countries can be as high as 30% [16]. Infertility has become one of the three diseases with the highest incidence. The high failure rate of assisted reproduction is caused by an important factor, which is ER [17]. The individual fertility is affected by many factors, such as hormone levels, ovarian functions, fallopian tube patency, and age. Under the circumstances, there is no significant difference in the above factors that can be monitored, and the success of conception depends on the level of ER [18]. With normal ER, we can successfully complete the process of fertilized egg implantation, implantation, angiogenesis, and placenta formation, so that there is normal growth and development of embryos.

As ER has been paid more attention, it has gone through a long time from what it is to how to promote it [19]. Through unremitting efforts, there are many methods to evaluate ER at present. Immunohistochemical detection at molecular level is the most accurate and the most recognized “gold standard” for evaluating ER. In recent years, the research on molecular biological mechanism related to ER has increasingly become the focus of attention [20]. However, biopsies are needed in molecular biology research. Because of its invasiveness, high price, and high requirements for laboratories, the scope of molecular biology research is greatly limited. Therefore, another popular research is the noninvasive, economical, and easily accepted method to evaluate ER.

Serological tests such as estrogen and progesterone have been widely employed in ART, while transvaginal ultrasound is more widely employed [21]. It is increasingly found that ultrasound can not only be employed to monitor ovulation, and many researchers and clinical workers in reproductive centers try to use ultrasound to evaluate ER, because this method is operable, noninvasive, convenient, and economical to benefit more patients. Abundant endometrial blood flow during the “window period” of implantation is a necessary condition for the endometrium to accept embryo reception. During this period, abundant neovascularization and good blood perfusion are the premises of ER [22]. More scholars have turned their attention to the blood flow parameters measured by transvaginal ultrasound, which are operable, economical, and easy to be accepted by the public, while which parameters of subendometrial blood flow have high value in the evaluation of ER.

Due to the lack of some performance of early ultrasound instruments, most of the previous studies focused on the blood flow parameters of the uterine artery, but the parameters of the uterine artery were not completely related to the parameters of subendometrial vessels and were affected by vascular resistance, blood flow velocity, and other factors [21, 22]. Gizzo et al. concluded in a recent study that the blood flow parameters of the uterine artery could evaluate the natural cycle but could not predict the stimulation cycle and endometrial blood flow without drug treatment [23]. However, another study pointed out that uterine artery blood flow parameters had nothing to do with pregnancy outcome, so it was impossible to predict pregnancy rate and had no practical value in evaluating ER [24]. Ahuja et al. found that the related indexes such as VI, FI, and VFI of endometrial blood flow in pregnant women were significantly higher compared to nonpregnant women and pointed out that endometrial blood flow parameters were an effective predictor of pregnancy outcome [25]. Different scholars have different opinions, and even different studies of the same scholar obtain completely different results, which make people confused about whether subendometrial blood flow parameters can predict ER.

In this study, the differences of type I and type III in late proliferation and type II and type III in ovulation period were statistically significant, indicating that transvaginal ultrasound could provide a certain reference for clinical observation of intimal and subintimal blood perfusion. The AUC and Pi values of the endometrium in the late proliferation and ovulation stage in the observation group were lower compared to those in the control group, while the AUC and Pi values in the observation group were significantly higher compared to those in the control group, and the difference was statistically significant. The results indicated that the blood perfusion of the endometrium and subendometrium in the late proliferation and ovulation stage control group was significantly better. Once the real implantation occurs, the endometrium changes to provide the necessary support for implantation, which is significantly different from that without implantation, and the lack of endometrial blood supply in front of the implantation window can lead to a decrease in ER.

Mature female ovaries reduce the ability to produce eggs and the quality of follicles, resulting in a decrease in fertility and sex hormones, which is called decreased ovarian reserve function (DOR). According to etiology, DOR can be assigned into nonphysiological DOR and physiological DOR, the former is not related to age, and the latter is related to age [22]. The former includes the following two types of women: (1) the etiology clearly causes the decline of ovarian reserve function, such as space-occupying lesions or after ovariectomy; (2) the etiology is unknown and the ovarian reserve decreases in patients younger than 35 years old. The latter means that the fertility of women decreases with age, mainly due to the decrease in the quality of eggs and the number of follicles left in the ovaries [23]. With the increase of female age, the number of follicles decreases and the quality of oocytes decreases, resulting in low fertility function, also known as low ovarian reserve function. Clinically, the commonly used methods to evaluate ovarian reserve function are anti-Mullerian hormone, basic hormone levels, which can accurately and quickly evaluate ovarian reserve function, but there is a certain degree of fluctuation in the menstrual cycle, which affects the test results. Three-dimensional transvaginal ultrasound technology uses a high-frequency probe to obtain high-definition images of pelvic organs, which can measure OV and AFC. AFC is the basis of mature follicles and can well reflect the number of primordial follicles in the ovary. According to relevant epidemiological studies [24], abnormal follicular development is the most common cause of female infertility, as high as 15% to 25%. Abnormalities in any link of the hypothalamus-pituitary-ovary axis will affect women's ovulation function, and ovulation has a direct impact on fertility results, so monitoring follicular development and detecting ovulation is an important problem in solving infertility. Basic body temperature and hormone levels are commonly used in clinical practice to evaluate the ovulation time of patients. Although the method is simple and easy to operate, it cannot directly reflect the changes of follicular morphology, lack of accuracy, and limitations. Transvaginal ultrasound can directly and clearly indicate the structure of the uterus and ovary [23, 24]. Considering abdominal B-ultrasound, it is not affected by pelvic organs, obesity, and other factors and does not need to fill the bladder. It is of great significance to treat infertility by monitoring follicular development, observing its maturity, finally judging whether ovulation, determining the cause of infertility, and then targeting treatment according to the results.

The results indicated that the levels of EDV, OV, AFC, and PSV in the normal response group were higher compared to those in the low response group, while the levels of FSH and FSH/LH in the normal response group were lower compared to those in the low response group, but the levels of LH and E2 were higher compared to those in the low response group [23]. Some studies have indicated that ovarian size reduction is related to ovarian aging [24]. OV < 3 cm has a lower response to ovulation induction and a higher rate of pregnancy failure. AFC can evaluate ovarian reserve function, because there are significant differences in the response of AFC in different ovaries, so it can not only judge the low response of the ovary but also be helpful for the diagnosis of ovarian hyperstimulation syndrome. The absence of AFC and the small size of the ovary suggest anovulation. According to the study of Ahuja et al., transvaginal Doppler ultrasound observation of ovarian hemodynamics can predict ovarian ovulation induction response [25]. PSV and EDV are closely related to ovarian response and can be used to predict ovarian response, so transvaginal Doppler ultrasound can predict ovulation and evaluate ovarian reserve function.

At present, the commonly employed clinical indicators to evaluate women's ovarian reserve function generally include two aspects: hormone level determination and ultrasound examination; the former includes follicle-stimulating hormone (FSH), basic E2, FSH/LH, inhibin B (INHB), and anti-Mullerian hormone (AMH); the latter includes AFC, OV, and ovarian interstitial blood flow [26]. FSH is a protamine hormone secreted by the pituitary gland, which can promote follicular development and maturation. Together with LH, it can promote the secretion of estrogen and cause ovulation. The increase of FSH level indicates premature ovarian failure. Basic E2 is produced by antral follicles, and the accuracy of predicting low ovarian response and pregnancy failure alone is very low. Fragouli et al. have proposed that there is no significant correlation between basal E2 content and ovarian response, so it is impossible to evaluate the ovarian response and ovarian reserve function. The pituitary secretes a variety of hormones, FSH and LH belong to two of them, and their function is to regulate ovarian function [27]. In the early stage of the decrease of female ovarian reserve function, the level of LH decreased, the level of FSH increased, and the ratio of FSH/LH increased; if the female ovary was in a state of failure, serum FSH and LH increased. Zhu et al. have indicated that when the FSH/LH ratio is ≥2, the quality of embryos, the number of eggs obtained, pregnancy outcome, and fertilization ability can be predicted for women aged between 35 and 37 years old [28]. Therefore, it is of high value in predicting ovarian function. The functional status of the hypothalamus and ovary can be indirectly understood by measuring the levels of FSH, FSH/LH, LH, and E2, which is helpful to predict the time of ovulation and evaluate the function of ovarian reserve. The results of this study indicated that FSH was negatively correlated with E2, EDV, OV, AFC, and PSV but positively correlated with FSH/LH. ROC curve analysis indicated that the cutoff values of EDV, OV, AFC, and PSV were 4.140, 3.725, 4.105, and 13.945, respectively, the specificity of each index was higher than 90%, and the sensitivity was higher than 80% except PSV. Among them, the AUC of AFC is the largest, so the ultrasound parameters of ovarian reserve function of AFC can be employed to predict the best index of ovulation, which is also confirmed by Jin Jing's study [28].

This study may also have disadvantages such as poor sample representation, inappropriate control selection, and bias in recall of exposure history. However, we tried our best to avoid them during the study to obtain reliable results.

Conclusively, three-dimensional transvaginal ultrasound can quantitatively analyze the microperfusion of the endometrium and subendometrial blood flow, provide the quantitative analysis index for clinical evaluation of uterine receptivity, and offer reference for clinical diagnosis and treatment; in addition, three-dimensional transvaginal ultrasound can also directly observe follicular development and monitor ovulation, which is of high value in evaluating ovarian reserve function and predicting ovulation.

## Figures and Tables

**Figure 1:** Comparison of blood perfusion types of the endometrium and subendometrium between the two groups.

**Figure 2:** Comparison of basal hormone levels between the normal response group and the low response group.

**Figure 3:** Ultrasonic parameters of ovarian reserve function and ROC curves of various indexes predicting ovulation.

**Table 1:** Comparison of the intimal AUC value and Pi value between the two groups ($\overset{¯}{x}\pm s$).

Group	*N*	Late stage of proliferation		Ovulation period		Planting window period	
		AUC	Pi (dB)	AUC	Pi (dB)	AUC	Pi (dB)
O group	308	184.39 ± 124.73	3.87 ± 1.72	142.17 ± 97.44	3.26 ± 1.55	167.55 ± 83.28	4.19 ± 1.85
C group	300	237.55 ± 119.73	5.64 ± 1.44	190.18 ± 103.26	4.97 ± 1.54	178.59 ± 84.26	5.34 ± 1.82
*t*		5.359	13.740	5.898	13.643	1.625	7.725
*P*		<0.05	<0.05	<0.05	<0.05	>0.05	>0.05

**Table 2:** Comparison of the subintimal AUC and Pi values between the two groups ($\overset{¯}{x}\pm s$).

Group	*N*	Late stage of proliferation		Ovulation period		Planting window period	
		AUC	Pi (dB)	AUC	Pi (dB)	AUC	Pi (dB)
O group	308	369.23 ± 179.18	8.65 ± 2.14	358.21 ± 152.17	6.44 ± 1.53	329.15 ± 134.28	7.27 ± 2.08
C group	300	307.22 ± 184.38	6.55 ± 2.07	297.54 ± 150.38	5.26 ± 1.48	345.36 ± 133.19	7.17 ± 2.44
*t*		4.206	12.294	4.495	9.662	1.494	0.544
*P*		<0.05	<0.05	<0.05	<0.05	>0.05	>0.05

**Table 3:** Comparison of general clinical data between the normal response group and the low response group ($\overset{¯}{x}\pm s$).

Group	*N*	Age of menarche (years)	Age (years)	Body mass index (kg/m^2^)	Menstrual cycle (d)
Normal response group	182	13.63 ± 2.34	35.24 ± 5.46	22.38 ± 3.32	27.73 ± 3.24
Low response group	126	14.15 ± 2.11	34.36 ± 5.63	22.43 ± 3.76	28.37 ± 3.25
*t*		0.204	1.470	0.131	1.826
*P*		>0.05	>0.05	>0.05	>0.05

**Table 4:** Comparison of the results of vaginal three-dimensional ultrasound between the normal response group and the low response group ($\overset{¯}{x}\pm s$).

Group	*N*	EDV (cm/s)	OV (cm^3^)	AFC (units)	PSV (cm/s)
Normal response group	182	6.28 ± 1.55	4.37 ± 0.76	6.24 ± 1.37	15.38 ± 3.65
Low response group	126	2.79 ± 0.76	2.87 ± 0.58	3.18 ± 0.43	9.66 ± 2.37
*t*		26.008	20.386	27.255	17.007
*P*		<0.01	<0.01	<0.01	<0.01

**Table 5:** Comparison of ultrasonic parameters of ovarian reserve function and indexes for predicting ovulation.

Variable	AUC area	Cutoff	Sensitivity	Specificity	Asymptotic 95% confidence interval
EDV	0.977	4.141	95.51	94.96	0.958~0.996
OV	0.954	3.726	83.22	95.81	0.934~0.977
AFC	0.983	4.106	93.33	99.17	0.968~0.998
PSV	0.885	13.944	62.64	99.19	0.846~0.921

## Data Availability

No data were used to support this study.
